The article "Reduced Gain and Shortened Time Constant of Vestibular Velocity Storage as a Source of Balance and Movement Sensitivities in Gravitational Insecurity" was published in 2022. Journal: Occup Ther Int.

# Reduced Gain and Shortened Time Constant of Vestibular Velocity Storage as a Source of Balance and Movement Sensitivities in Gravitational Insecurity

**DOI:** 10.1155/2022/5240907

**Published:** 2022-05-06

**Authors:** Michael Potegal, Teresa A. May-Benson, Sara Oxborough, Amy Hall, Stefanie McKnight

**Affiliations:** ^1^University of Minnesota, USA; ^2^Spiral Foundation, USA; ^3^National Dizzy and Balance Center, USA

## Abstract

Gravitational insecurity (GrI) involves lifetime movement and balance concerns whose pathophysiological origins are unclear. We tested whether balance symptoms in mild GrI might involve anomalies in vestibular velocity storage (VVS), a brainstem/cerebellar circuit that amplifies gain and prolongs the persistence of weak vestibular signals from small/slow head movements. A Provisional Gravitational Insecurity Index (PGrI) was developed, evaluated for psychometrics/demographics, and used to identify otherwise healthy adults with life-long balance challenges as well as sex, age, and ethnicity-matched comparison adults without such challenges. Balance confidence, sensory hypersensitivities, spatial orientation, anxiety, and hearing loss were self-reported. Standing balance under visual/proprioceptive restrictions and perrotary vestibulo-ocular nystagmus were evaluated. The PGrI showed approximated test-retest reliability and convergent and discriminant validity. When only vestibular input was available, mild GrI participants on a tilting platform used effortful hip strategies for balance significantly more than did comparison participants. Rotation testing revealed that mild GrI participants had significantly less low frequency gain and shortened VVS persistence. Combined, these two parameters correlated significantly with PGrI. The PGrI also correlated with problematic spatial orientation, but surprisingly, not to anxiety. Balance/movement issues in GrI are likely due to VVS deficiencies. Additional mechanisms may account for other GrI symptoms. Better understanding of GrI's pathophysiological basis will be useful in informing the larger health-provider community about this condition.

## 1. Introduction

Occupational therapists trained in Ayres Sensory Integration® (ASI) theory routinely assess and treat individuals who hesitate, fear, and avoid movement activities requiring balance such as standing on one foot, being on an unstable or moving surface, or maintaining body stability when leaning over to perform instrumental activities of daily living. These are characteristic symptoms of gravitational insecurity (GrI), which is classified as a sensory modulation problem due to the associated emotional reactions and has been attributed to otolith organ dysfunction. However, most of what is known about GrI comes from its presentation in childhood as a reluctance to move the head out of an upright orientation (e.g., to lay back or somersault), sensitivity to motion (e.g., turning corners in cars), and fear of losing balance (e.g., on uneven or yielding surfaces or playground equipment [1]). These children often refuse to climb, swing, skate, or bike and may be teased about their clumsiness and/or nonparticipation in sports. May-Benson and Koomar's [1] validation of behavioral measures for identifying GrI in American 5-10 year olds was cross-culturally confirmed in Indian 3-9 year olds [2]. Potegal et al. [3] raised questions about the typically extensive motor and emotional comorbidities in childhood GrI which they provisionally resolved in favor of GrI being a distinct nosological entity with its own presumptive pathophysiology based on a small number of cases in which the movement and balance symptoms of GrI presented in isolation.

Childhood GrI can continue into adulthood, per May-Benson et al.'s [4] finding that 2% of a normative sample of 1,392 adolescent and adults reported avoiding head positions out of the upright when driving or hair-washing, great fear of falling on slippery, moving or unstable surfaces and climbing chairs/ladders, and a compelling need to “keep their feet on the ground,” as they say about themselves (cf., [5]). An additional 17% presented with mild GrI, i.e., similar but less severe symptoms of caution and anxiety when facing these challenges. However, less is known about these adult forms of GrI.

Contemporary neuroscience does recognize a reciprocal association between anxiety and imbalance [individuals with balance problems are more likely to be anxious, anxious people are more likely to have balance problems e.g., [6]. From a neuroscience perspective, the fear-inducing movement and balance-related problems of adults with GrI could arise from abnormal processing in one or more of three sensory systems that control movement and balance: proprioceptive signals about joint angles and limb positions, whole visual field optic flows that signal self-movement through space, and vestibular input. Standard clinical posturography on a sway platform is routinely used to evaluate the function of these sensory systems [7]. Besides assessing sensory control, posturography can identify when people struggling to maintain their balance switch from using postural adjustments around the ankles to faster but less efficient and more effortful adjustments around the hips. In this study, we analyzed balance strategies of adults with mild GrI with posturography to better characterize this condition.

Childhood GrI symptoms do overlap with classic vestibular signs [3], supporting proposals that GrI involves some form of vestibular dysfunction [8, 9]. If so, GrI cannot be due to anomalous otolith signals alone, as some have suggested [9], because labyrinth biophysics dictates that the otolith organs by themselves cannot distinguish between head tilt (orientation to gravity) and linear acceleration. Discrimination of how the head is actually moving requires moment-to-moment signaling of tilt rotation by the semicircular canals [10]. However, semicircular canal biophysics results in signals from small and/or slow head rotations that are, by themselves, too weak and too short for adequate discrimination of such movements. These low frequency signals are, therefore, amplified and prolonged by a brainstem/cerebellar vestibular velocity storage (VVS) circuit that integrates canal signals over time [11]. We conjectured that individuals with GrI may need to maintain a stable upright head orientation as they move because an inadequate VVS signal impairs their ability to adequately discriminate head tilt from linear acceleration. The VVS circuit is distributed among the anterior part of the medial vestibular nucleus, vestibular commissure, and cerebellar nodulus [12]. Thus, as suggested by May-Benson and Koomar [1], dysfunction of central vestibulo-cerebellar circuits may be involved in GrI.

Gain (amplification) and time constant (persistence) of nystagmus in the dark are relevant VVS parameters that are routinely measured during clinical diagnosis of peripheral or central vestibular (dys)function. For example, shortened VVS time constants have been found in fall-prone older individuals [13] and in adults self-identified with some combination of clumsiness, movement intolerance, gravitational insecurity, and “vestibular system dysfunction” [14]. Conversely, excessively prolonged time constants are associated with motion sickness [15], migrainous vertigo [16], and Meniere's disease [17]. Based on observations that nystagmus durations in children with GrI were sometimes shorter but often longer, Ayres and Robbins [8], p. 85] proposed that GrI might be associated with prolonged durations. Theory does suggest that VVS output could become unstable if the time constant is too prolonged [18]. Thus, GrI pathophysiology might involve time constants that are either too short or too long. Fortunately, standard clinical rotation-test diagnostics yield reliable estimates of VVS gain and time constant parameters to resolve the question of time constant duration.

The multiple comorbidities that often present with GrI are another issue from a neuroscience perspective. While fear of movement is a defining characteristic of GrI, fine and gross motor difficulties and anxiety are the three most commonly associated problems reported by pediatric OTs [3]. Less is known about GrI comorbidities in adulthood. It is unclear if general anxiety is characteristic in adult GrI or if their discomfort is specific to movement/balance challenges. Clinical observations do suggest that emotional reactions to movement/balance challenges in adults with mild GrI amount to hesitancy and discomfort rather than the intense fear seen in children [19]. Various sensory hypersensitivities also co-occur with adult GrI [4]. Additionally, anecdotal reports of impaired direction sense associated with GrI might be due to defective VVS input to the parietal cortex, hippocampus, and/or basal ganglia, which use such input for inertial navigation through space [20, 21]. Vestibular dysfunction can be associated with hearing loss [22], which was assessed by self-report.

The present study is an occupational therapy (OT)—neuroscience collaboration on balance and vestibular (dys)function-related issues in adult GrI. However, adults with severe GrI are relatively rare in OT clinics and often find rotary testing too distressing. Thus, individuals with milder GrI (MGrI) symptoms are more likely to participate in testing. Furthermore, vestibular function declines with age [23], age by sex interactions have been reported for various vestibular conditions [24], and ethnic differences in balance and vestibular function occur across the life-span [25]. Similarly, vestibular problems, like other medical issues, are more prevalent in lower socioeconomic/educational (SES) groups [26]. Hence, matching individuals with mild GrI symptoms beginning in childhood to a non-balance challenged typically functioning comparison group within these categories is necessary for the most valid resolution of these issues. Specific aims of this study were to: (1) posturographically assess balance strategies used by individuals with a life history of GrI symptoms, (2) determine if anomalies in vestibular velocity storage (gain and/or time constant) relate to GrI symptoms, and (3) identify which comorbidities are associated with such histories.

## 2. Materials and Method

This study had two separate parts. First, a screening measure was developed using survey methodology to identify adults with a history consistent with MGrI and sex, age and ethnicity-matched individuals with no such history. Second, participants' visual, proprioceptive, and vestibular control of balance was assessed with diagnostic posturography. Their vestibulo-ocular response to rotation was then evaluated to assess VVS gain and time constant. Finally, to identify the functional profile of adult GrI comorbidities, screening scores were correlated with participants' self-report of direction sense, sensory hypersensitivities, and anxiety. University of Minnesota IRB approval was obtained (STUDY00002249); written consent was obtained from all participants.

### 2.1. Provisional Gravitational Insecurity Index (PGrI) Development

Based on informal but detailed interviews with adults reporting GrI signs and OTs' experience with such individuals, eight items from the vestibular processing scale of the *Sensory Profile Caregiver Questionnaire* [27] and the movement processing scale of *Adolescent/Adult Sensory Profile* [28] that were most germane to the information provided were selected and reworded to be consistent with adult recall of childhood movement experiences (Table 1). Response options were reformatted as “bothered me not at all,” “a little,” or “a lot” [29]; respective scores of 0, 1 or 2 produced an PGrI index score range of 0-16.

### 2.2. Survey Respondents

The PGrI index was completed by 112 University of Minnesota OT Masters or Doctoral students and staff of Twin Cities OT clinics (104 female, *M* = 26 ± 5 yrs) and 90 visitors to the OT booth at the Minnesota State Fair 8/22/2019 (57 female, *M* = 57 ± 13 yrs). Visitors completing the PGrI were given a souvenir pen. Survey respondents noted sex and age but were otherwise anonymous. For clinical comparison, seven adults with GrI and 10 without GrI, as identified by the *Adult/Adolescent Sensory History* (ASH, [30]) in a large northeastern OT facility also completed the PGrI (sex and ages not given per IRB deidentification requirements). These 17 clinical survey respondents were not tested in the laboratory study.

### 2.3. Study Participants

Participants with symptoms characteristic of mild GrI since childhood were recruited through flyers posted around University of Minnesota, on community bulletin boards and Twin Cities yoga studios as well as by word-of-mouth through OT Masters students. Responders to study notices were interviewed by telephone to complete the PGrI and review exclusion criteria. Exclusion criteria included report of >1 concussion, any neurological injury or disease, and a history of migraines or vertigo. Responders with clinical level PGrI scores ≥ 7, per Figure 1, were emailed a copy of the consent form to review. If consent was given in a follow-up phone call, they were recruited into the GrI group (written consent was obtained in person before the testing began).

A modified case-control recruitment matched the GrI study group to comparison participants by age, sex, and ethnicity. Individuals screened into the GrI group nominated relatives, friends, and community acquaintances who had consented to be contacted by the first author. When necessary, local OT and other communities were contacted for matches by sex, age (±6 yrs), and ethnicity. Per Figure 1, matching individuals with PGrI scores ≤ 3 (i.e., from the 70% of the population with least balance problems) were recruited into the study comparison group. Participants were asked about their highest level of education as the most common, least intrusive SES measure [31]. All study participants were compensated $50 for their time.

The 34 participants who completed testing included 14 Caucasian matched pairs, 2 Asian pairs, and 1 African-American pair (three would-be participants did not complete testing). Twelve of the 17 completing pairs were female. Participants were 20–70 years old. The case control matching resulted in equivalent years of education (Table 2).

### 2.4. Measures

#### 2.4.1. Self-Report Interview and Questionnaires

A structured interview was completed with each participant that included current adult experience of care taken while walking under different conditions (0 to 3 scale), level of hearing disability and eight movement activities that were the adult equivalent of the items on the PGrI. (Six of these items are interchangeable with the 9 item subset of questions about movement/vestibular processing on the ASH that are used to identify clinical-level adult GrI). Participants also recalled childhood events that might be associated with GrI including their least preferred sleeping position (on stomach, back, or side; difficulties with athletic activities/sports and history of falls [3]. Participants also completed the following standardized scales: *Activities-Specific Balance Confidence Scale* (ABC, [32]), *Santa Barbara Sense of Direction Scale* (SBSOD, [33]), *Sensory Over-Responsivity Scales* (SOR, [29]), and the *State-Trait Anxiety Inventory* (STAI, [34]).

#### 2.4.2. Posturography

The Equitest dynamic posturography machine (Neurocom Inc, v8.0, 2001) measures maximum body sway amplitude during three 20 sec trials under each of six sensory conditions [7]. In the “proprioception” condition ankle proprioception for balance control is eliminated by tilting the floor plate to keep ankle angle constant as the body sways. In the “visual” condition, wall tilting that keeps visual distance to the wall constant eliminates optic flow. Ankle proprioception and optic flow are both eliminated in the “vestibular” Condition, so balance is under vestibular control. Score ratios for different combinations of the six conditions yield percent scores for proprioceptive, visual, and vestibular control of balance.

People using compensatory hip strategies of balance create shear force oscillations that are transmitted through their feet to the floor plate. These oscillations appear as episodes of distinct high frequency waves in trial records. Oscillation frequency, amplitude and percent duration were measured on enlarged printouts of each trial record. In trials terminated by a loss of balance, force, frequency and percent duration of oscillations before balance loss were calculated and used.

#### 2.4.3. Vestibular Function Tests

Gains and time constants of vestibulo-ocular response to rotation was measured using a motor-driven, computer-controlled rotary chair (Neuro Kinetics, Inc. VEST™ V6.8 Chair Controller). An infrared camera (Neuro Kinetics, Inc. I-Portal-VOG® V.2.4.002 4D Video-Oculography System) recorded the eye movements of per-rotary nystagmus. Following standard clinical diagnostic protocols, individuals were tested under four conditions with two to four trials per condition: (1) visual suppression test of visual-vestibular interaction in which participants was rotated back-and-forth in sinusoidal harmonic acceleration (SHA) for 18 sec at .16 and .32 Hz while fixating on a light attached to the chair, which normally suppresses nystagmus; (2) visual enhancement test in which a stationary light pattern projected on test chamber walls during SHA added optokinetic stimulation to the experienced rotation, normally enhancing nystagmus; (3) cycles of SHA at frequencies of .01, .04, .08, and .16 Hz in the dark (VVS function is predominant at .01 Hz); and (4) clockwise/counterclockwise velocity step tests in which the chair rapidly accelerates to 60°/sec angular velocity which is then maintained for 45 sec. Gain in per-rotary nystagmus was measured in all tests while VVS time constants were measured only in the step test.

### 2.5. Data Analyses

Data were analyzed as follows: (1) PGrI demography (percents of population represented by GrI and comparison group score ranges), (2) PGrI reliability and validity (correlations with standardized scales and group differences), (3) group differences in posturography (maximum sway and shear force oscillation), (4) group differences in vestibular function (gain and time constant) using ANCOVAs with age as covariate, and (5) PGrI comorbidity profile (PGrI correlations with the four standardized questionnaires).

## 3. Results

### 3.1. PGrI Demographics

A Kolmogorov-Smirnov test of pooled younger and older survey respondent data found a significant shift to higher PGrI scores in females versus males (*D* = 0.25, *p* < .03). Comparing study groups' PGrI scores to the survey scores distribution, the comparison group represented a sample from the 70% of the population with fewest balance problems. The MGrI group was selected from people above the 91^st^ percentile for PGrI index score, comparable to individuals with clinically identified GrI (Figure 1).

#### 3.1.1. PGrI Index Reliability

Test-retest reliability of the PGrI was approximated by comparing scores from the telephone administration of the eight childhood experiences in Table 1 to the test-site scores for eight adult experiences obtained 28 ± 20 days later. Approximated test-retest reliability was high (*r* = 0.90, *p* < .001).

#### 3.1.2. PGrI Index Validity

Convergent validity of the PGrI index was demonstrated by significant correlation with the *ABC Scale* (*r* = −.73, *p* < .001). Discriminant validity was evident from the significantly greater caution reported by MGrI participants when walking than the comparison participants (Table 2). Additional approximations to discriminant validity and clinical relevance of the index were indicated by higher PGrI scores of 7 adults in an OT clinic identified with GrI (range 4-14) versus 10 adults in the clinic identified as not having GrI (range 0-2, Mann–Whitney *U* = 70, *p* < .001). See Figure 1.

### 3.2. Posturography

As expected, all participants swayed progressively more widely under proprioceptive, visual, and vestibular conditions, per a pairwise repeated measures ANCOVA with age as a covariate [*F*(2, 13) = 6.47, *p* = .005]. There were no between-group differences in maximum sway. However, there were differences in shear force oscillation. Overall, the MGrI group had significantly more forceful, higher frequency and longer duration shear force oscillations than the comparison group in the vestibular condition. This indicated greater MGrI reliance on more effortful hip strategies versus ankle strategies when balance was challenged and they had only vestibular inputs to rely on [repeated measures ANCOVA *F*(1, 13) = 7.4, *p* < .02]. See Table 2 for individual variable values.

### 3.3. Vestibular Function Parameters

Consistent with previous reports [23], the comparison group showed reduced step gain and mean SHA gain with age (*r* = −.47 and − .53 and *p* < .05, respectively), thus justifying the use of the matching protocol as well as age as a covariate in statistical analysis. A repeated measures MANCOVA with age as covariate showed no between-group differences in visual suppression or visual enhancement [*F*(1, 14) = 2.9, NS], indicating that MGrI balance symptoms are not due to aberrant visual-vestibular interaction. Crucially, the MGrI group showed less robust function than the comparison group in both vestibular parameters. A repeated measures ANCOVA found that the MGrI velocity step per-rotary time constant was significantly shorter [MGrI *M* = 12.8 ± 4.9 sec, comparison *M* = 16.5 ± 5.0 sec; *F*(1, 14) = 6.44, *p* = .024]. As Figure 2 shows, MGrI gains were somewhat higher at SHA frequencies above .01 Hz. However, a second ANCOVA found MGrI gain was significantly lower than the comparison group [MGrI *M* = 0.4 ± 0.1, comparison *M* = 0.45 ± 0.12; *F*(1, 14) = 6.2, *p* = .026] at SHA .01 Hz, the frequency at which VVS contributes most strongly to vestibular performance.

To assess the association between the PGrI and the two vestibular parameters that distinguished the groups, the .01 Hz SHA gains and velocity step time constants for all subjects were converted to Z scores. Mean combined Z scores were then calculated. After removal of two clear outliers, the correlation between PGrI and mean combined vestibular parameter Z scores was significant (*r* = −0.56, *p* < .001).

### 3.4. Spatial Orientation, Sensory Hypersensitivity, Anxiety, and Hearing

Scatterplots of Santa Barbara Scale data showed that increasing PGrI correlated significantly with decreasing spatial orientation skills both within and across groups (overall *r* = −0.48, *p* < .001). The PGrI to SOR correlation was significant across groups (*r* = .39, *p* = .024), but this was due to the MGrI group's slightly higher mean SOR score. There were no significant within-group correlations of SOR score with the PGrI (*r* ≤ .31, NS). Anxiety was uncorrelated with PGrI scores (*r* = 0.1, NS). Seven participants in the MGrI group and two in the comparison groups self-reported at least mild hearing impairment; this difference was not statistically significant.

### 3.5. High Sensory Hypersensitivity MGrI Subset

MGrI group participants with the highest SOR scores, which reflect the greatest overall sensory hypersensitivity, were more likely to report each of three markers of childhood GrI: dislike of sleeping on the back, falling more than other children and being teased about clumsiness and sports nonparticipation. The five MGrI individuals with the highest SOR scores, 30% of that sample, accounted for 57%-75% of all those reporting each marker. These asymmetries in childhood GrI marker distributions within the MGrI group were highly statistically significant by Shapiro-Francia [35] normality tests (W′s > .21, *p* < .001). However, the MGrI group SOR scores were unrelated to their PGrI, anxiety scores, or the combined vestibular parameter Z score, suggesting that sensory hypersensitivity is not intrinsic to mild GrI.

## 4. Discussion

Several reported findings substantiate study method validity and credibility of results. Thus, female respondents in the PGrI survey reported more balance difficulties as children than did males, consistent with May-Benson et al. [4], Potegal et al. [3], and sex differences in vestibular function and fall risk [36]. The age ranges and percentages of female survey respondents were comparable to those of study participants. Our confidence that study participants selected for mild GrI were appropriately identified is bolstered by the equivalence of items on the adult form of the PGrI with the ASH clinical diagnostic movement/vestibular processing items as well as by the clear overlap of their PGrI scores with those of adults clinically identified with GrI, as shown in Figure 1. Methodological strengths include matching MGrI and comparison participants for sex, age and ethnicity that resulted in comparable years of education as an SES measure. Movement/balance related symptoms retrospectively self-reported in the PGrI, the stepping caution question and ABC scale were confirmed by objective observation of increased hip strategy usage by the MGrI group during posturography testing. There were no group differences in postural sway, but the MGrI group used more hip strategy in the vestibular condition providing evidence that, when using only vestibular input, they had to exert more effort than the comparison group to maintain the same level of balance.

Several lines of evidence suggest that movement/balance-related symptoms associated with GrI originate centrally rather than in the inner ear. Inner ear dysfunction was made less likely as a symptom cause because individuals with a history of vertigo were excluded and group differences in self-reported hearing impairment were not statistically significant. Rotation testing found no difference between groups in visual suppression or enhancement of vestibulo-ocular reflexes, suggesting that the pathophysiology that generates GrI is not on the input side but within brainstem/cerebellar vestibular circuitry. Rotation in the dark revealed a combination of reduced low frequency gain and shorter time constants (i.e., shorter nystagmus durations) that together correlated with GrI severity. Thus, a less robust VVS signal may well cause some of the movement/balance symptoms in mild GrI. These results are entirely consistent with Fisher et al. [14] whose self-identified vestibular dysfunction group had significantly shortened per- and postrotary velocity step time constants and also longer phase lags at .01 Hz SHA, but not at higher frequencies. Longer phase lags are associated with shorter time constants. Thus, anomalies of velocity storage in vestibulo-cerebellar circuits may be a key pathophysiology in GrI.

Anecdotal reports of spatial disorientation associated with GrI were also confirmed. To the extent that VVS signals ascend to brain structures that track direction and distance of self-movement, anomalous VVS signals would make moving through the environment disorienting and way-finding difficult [20, 21].

The PGrI scores of the MGrI group fell within the lower end of the range of the OT clinic adults identified with GrI, so these results apply to mild GrI. There was no significant relationship between anxiety and GrI symptoms, suggesting that GrI-related discomfort is specific to movement/balance challenges and not general anxiety, consistent with May-Benson et al. [4, 19]. That is, the balance, hypersensitivity, and anxiety aspects of GrI appear to be partially independent of each other; adults with GrI may experience varying levels of each.

These interpretations of results in no way challenge routine observations of multiple comorbidities of core movement/balance-related symptoms in individuals with full-blown GrI seen in OT clinics. Nor do they challenge the proposition that some comorbidities reflect hyperreactivity to various sensory stimuli. The question of how these comorbidities arise remains. It may be that individuals with multiple issues are more likely to seek professional help than those with mild challenges, so present with a larger range of more serious problems. Additionally or alternatively, the VVS anomalies that cause GrI and its associated comorbidities might arise from different processes. For example, the VVS is replete with B type receptors for the powerful inhibitory neurotransmitter GABA [12]. The shortening of the VVS time constant by the GABA-B agonist baclofen (Lioresal) confirms the importance of these receptors for balance [37]. But, GABA B receptors are practically ubiquitous in the brain, including in anxiety-mediating structures [38]. So, a defect in the GABA B gene on chromosome 6 might well create vestibular dysfunction that correlates with a range of otherwise unrelated behavioral problems. That is, the various behavioral signs of GrI correlate merely because GABA B receptors happen to play a role in a number of independent and functionally unrelated neural circuits.

## 5. Limitations and Future Studies

Although our results replicate key findings of Fisher et al. [14] with twice their sample size, both are small N studies that need replication. VVS time constants decrease with up-tilt of the head [39] possibly explaining why people with GrI are distressed by and avoid tilting back, which would further reduce their already shortened time constant. If so, rotary testing of vestibulo-ocular reflexes with upward head tilts of, say, 45° might further clarify the VVS deficiency in GrI.

The finding of underpowered VVS in GrI does not eliminate the possibility that otolith organ signals are dysfunctional as well. Although hearing impairment did not differ significantly between the groups, the larger number of MGrI participants self-reporting such problems raises a question about inner ear function. Otolith organ input in GrI and controls could be easily compared with a purely visual rod-in-frame test [40]. An advantage of this test is that it is taken sitting down and involves no body or head motion, so might be amenable to people with more severe GrI.

## 6. Conclusions and Implications for Occupational Therapy Theory and Practice

OT intervention approaches should be developed around an understanding of VVS functions and features. Integrating an understanding of the VVS circuit and mode of operation into sensory integration theory and practice would be of benefit to practitioners and their clients. In clinical practice, clients with GrI and related conditions may present with varying combinations of movement/balance sensitivities, so therapists are encouraged to examine the individual constellation of client symptoms and comorbidities to best determine an intervention plan.

Alternatively, or additionally, OTs might consider reviewing and adopting some of the behavioral procedures and practices used in vestibular rehabilitation [41] in their interventions for GrI.

Underpowered vestibular velocity storage that generates a signal that is too weak and too short in GrI would seem to qualify as a sensory discrimination problem, but the discomfort that is specifically linked to movement/balance challenges in mild GrI suggests a sensory modulation problem. It might be worthwhile to rethink the theoretical categorization of GrI as discriminative-postural vs. modulatory-emotional, and perhaps the categories themselves, based on a deeper understanding of central vestibular physiology.

To date, GrI has been recognized almost exclusively by OTs. Based on an understanding of peripheral vestibular biophysics and central neurophysiology, our analysis found that the movement/balance symptoms in at least some individuals with mild GrI are associated with an underpowered VVS. In the context of general interprofessional clinical practice, these results should help introduce GrI to the larger health provider community to the credit of occupational therapists who have identified a hitherto unrecognized form of mild idiopathic bilateral vestibulopathy [42].

## Figures and Tables

**Figure 1:** Population, study, and clinic sample PGrI scores plotted on a modified log scale. Back row population sample (black, *N* = 202): 70% have scores ≤3 and 9% have scores ≥7. Upper right inset: linear *y*-axis number scale shows true left skew of population scores. Front row clinic sample: OT clinic individuals without GrI (white) and OT clinic individuals with GrI (gray). Middle row: study comparison group (vertical stripes) is from 70% of population without balance problems. Balance-challenged MGrI scores (horizontal stripes) are within range of OT clients with GrI.

**Figure 2:** MGrI and comparison group SHA and velocity step gains.

**Table 1:** Items from the Provisional Gravitational Insecurity Index.

	As a child, these kinds of activities bothered me (not at all, a little, a lot)
1	Climbing, like on ladders and jungle gyms
2	Climbing up or walking down stairs without a railing, like in an open stairwell
3	Experiencing heights, like a top bunk in a bunk-bed, being on a rooftop, top of a tall building, or tourist lookout
4	Walking on uneven surfaces, like a gym mat, beach sand, and forest trail
5	Standing or walking on moving surfaces, like in buses, trains, or on moving walkways
6	Using playground equipment, like swings and slides
7	Going on amusement park/state fair rides
8	Being lifted off the ground, like being picked up as a young child or going on Ferris wheels or ski lifts when older

**Table 2:** Demographics of the mild GrI and comparison groups; results of walking caution question and ANCOVAs of shear force oscillation measurements.

Group	Demographics		Results			
	Mean age (± SD)	Years of education	Walking caution (median, IQR)	Vestibular trial shear force oscillation		
				Frequency (Hz)	Force (lbs)	% duration
MGrI	38.5 ± 15.1	17.1 ± 2	1.5, 1-2	1.50 ± 0.94	5.68 ± 3.58	34.2 ± 30.6
Comparison	38.2 ± 14.1	16.9 ± 1.3	0, 0-0	0.93 ± 0.58	2.99 ± 2.73	19.4 ± 19.1
Test Statistic	*t*(16) = .26 NS	*t*(16) = .59 NS	Wilcoxon test *W* = 105, *p* = .001	*F*(1, 13) = 6.8 *p* = .02	*F*(1, 13) = 7.5 *p* < .02	*F*(1, 14) = 8.8 *p* = .01

Two bottom rows: ANCOVA values.

## Data Availability

Data are available from the first author.
